The article "Application of PDCA Circulation Regulation Combined with Nursing Mark in Nursing Safety and Quality Regulation of Disinfection Supply Center" was retracted in 2023. Reasons: suspected computer-generated content; unreliable results or conclusions; lack of ethics approval or compliance; missing or withdrawn patient consent.

# Application of PDCA Circulation Regulation Combined with Nursing Mark in Nursing Safety and Quality Regulation of Disinfection Supply Center

**DOI:** 10.1155/2022/9253777

**Published:** 2022-08-16

**Authors:** Xiuyu Cai, Jun Li, Wen Li

**Affiliations:** ^1^Central Sterile Supply Department of the First Affiliated Hospital of Hainan Medical College, Haikou 570102, China; ^2^Nursing Department of the First Affiliated Hospital of Hainan Medical College, Haikou 570102, China

## Abstract

**Objective:**

A case-control study was conducted to explore the application value of PDCA cycle regulation combined with nursing label in nursing safety and quality regulation in disinfection supply centers.

**Methods:**

The medical staff in the disinfection supply center of our hospital from January 2020 to December 2020 and from January 2021 to December 2021 were included in the control group (routine nursing regulation, *n* = 13) and the research group (PDCA circulation nursing regulation, *n* = 13). The differences in quality evaluation, disinfection qualification, quality regulation effect, supply satisfaction, job satisfaction, safety awareness, and comprehensive operation skills of nursing staff were compared, and the application value of PDCA cycle regulation combined with nursing label in nursing safety and quality regulation of disinfection supply center was comprehensively analyzed.

**Results:**

The quality score of nursing staff, and quality evaluation in the study group was significantly higher than that in the control group, and the difference was statistically significant (*P* < 0.05). The disinfection qualification rate of nurses in the research group was significantly higher, and the difference was statistically significant (*P* < 0.05). The effect of device quality supervision in the study group was significantly improved, and the difference was statistically significant (*P* < 0.05). The scores of various supervisions in the study group were significantly higher than those in the control group, and the difference was statistically significant (*P* < 0.05). The safety recognition ability, risk prevention awareness, service awareness, and theory and operation scores of nurses in the study group were significantly higher than those in the control group, and the difference was statistically significant (*P* < 0.05). The incidence of adverse events in the study group was lower, and the difference was statistically significant (*P* < 0.05). The satisfaction of the research group was significantly higher than that of the control group, and the difference was statistically significant (*P* < 0.05).

**Conclusion:**

In summary, the implementation of the PDCA cycle supervision method in the supervision of the sterile supply center in conjunction with the nursing logo is conducive to improving the quality of supervision and sterilization of all work aspects of the sterile supply center, reducing the occurrence of adverse nursing events and promoting the job satisfaction of nurses. In addition, it is conducive to standardizing the operational processes of staff, improving self-learning awareness enhancement, and improving work quality and efficiency.

## 1. Introduction

PDCA refers to the initials of Plan (plan), Do (implementation), Check (inspection), and Action (action), respectively, and is the scientific level followed by “total quality regulation” (TQM). Through PDCA cycle, the final aim of PDCA cycle regulation is to enhance the quality of service, product, or work step by step and optimize various work [1]. The disinfection supply center is responsible for the centralized regulation and treatment of reusable medical devices and articles in the hospital [2, 3]. As medical devices will come into contact with a large number of patients in the process of repeated use, and their surfaces are easy to retain bacteria to cause nosocomial infection, hospital disinfection and supply centers should strengthen their own work regulations. The staff of the disinfection and supply center should also do a good job of safety protection to ensure their own safety, while thoroughly controlling and eliminating the source of infection and ensuring the safety of users of medical devices [4, 5].

The quality of nursing regulation in the disinfection and supply center is directly relevant to the medical level of the hospital and the health of patients [6]. If the disinfection and supply center is not managed properly, or if the nurses do not have a strong sense of safety, it will lead to more serious medical accidents, which will not only be not conducive to the recovery of patients but also increase the medical expenses of patients, it has a serious adverse impact on the social image of the hospital [7]. Only nurses are strongly aware of the importance of nursing safety, can they carry out strict and serious disinfection and sterilization of the articles in the disinfection and supply center, and ensure medical safety [8]. At present, the nursing regulation of disinfection supply center puts more emphasis on nursing staff and nursing process. However, with the increase of hospital scale and equipment, the work burden of disinfection supply centers is getting bigger [9]. How to enhance the nursing efficiency and nursing quality of disinfection supply centers more effectively has become the focus of clinical research. Although nursing logo has long been adopted in disinfection supply centers, the traditional usage is mainly adopted for simple marking to distinguish. With the continuous development of clinical research, through clear nursing logo in improving the efficiency and quality of nursing care in disinfection supply centers has received widespread attention. Nursing signs are used to ensure the safety of clinical care, nursing care, and patients, and to ensure the smooth operation of nursing work, and are characterized by the use of standardized words and patterns to warn of work aspects in nursing work. In order to ensure the safe use of sterile items in the clinical setting and to improve clinical satisfaction, this study further explores the effectiveness of the application of nursing signs in the nursing safety management of disinfection supply centers.

PDCA cycle theory is a standardized and scientific cycle theory system put forward by Dai Ming, an American quality regulation expert, which can be applied to quality regulation [10]. It has become the basic method of nursing regulation. The PDCA cycle model summed up according to the objective law accords with the objective law of understanding things, that is, “practice-cognition-re-realization-re-cognition” is scientific. Since the 1980s, the regulation method of PDCA cycle theory has been introduced into the medical field [11, 12]. After popularization and application, it has been widely recognized in the industry. At present, the application of PACD cycle theory is more mature and has achieved good results in nursing quality regulation and other work. Bombard et al. use PDCA cycle quality regulation to remarkably reduce the risk of nosocomial infection, promote the infection control awareness of medical staff, and reduce occupational risks [13]. Realyvásquez-Vargas et al. used PDCA cycle to educate medical staff and medical staff in the hospital, and the behavior compliance rate and satisfaction of nursing staff and medical staff were remarkably enhanced [14]. Nsafon et al. effectively solved the clinical nursing problems through FOCUS-PDCA theory, improved the self-nursing ability of rectal cancer patients undergoing colostomy, and further confirmed that FOCUS-PDCA is a logical and accurate systematic regulation method [15]. There are many medical instruments in the hospital that need to be adopted repeatedly, especially some surgical instruments that are very sophisticated and valuable, and need to be carefully sterilized and preserved for use in reoperation. In January 2019, our hospital began to apply PDCA circulation regulation mode to the work regulation of disinfection and supply center, and the application effect is satisfactory, which is reported as follows:

## 2. General Information and Methods

### 2.1. General Information

The subjects of this study were 13 nurses in the disinfection and supply center of our hospital. The routine regulation method was implemented in the department from June to December 2019, and the PDCA cycle regulation method was implemented from January to June 2020. Among the 13 nurses, 13 were female, aged from 24 to 49, with an average age of (32.64 ± 3.29) years, 1 with college degree or less, and 12 with bachelor's degree or above.

### 2.2. Treatment Methods

The disinfection and supply center will implement the routine regulation method from January 2020 to December 2020, that is, to complete the recovery, classification, cleaning, disinfection, inspection, and storage of instruments and equipment according to the routine regulation system and process of the disinfection and supply center. The PDCA cycle regulation law will be implemented from January 2021 to December 2021, and the contents are as follows: (1) The planning stage. A PDCA cycle regulation team was set up under the leadership of the head nurse. According to the four working processes of recovery and classification, cleaning and disinfection, inspection and packaging, and storage and distribution in the disinfection supply center, all nurses were assigned into four groups, each group was led by senior nurses. Before the implementation of the PDCA cycle regulation method, the head nurse summoned the team members to analyze the problems existing in the current disinfection supply center and their causes, worked out the PDCA circulation regulation measures, and planned the regulation objectives of the disinfection supply center and the hospital infection control objectives according to the actual situation of our hospital; (2) The head nurse summarizes the regulation quality according to the relevant standards of each work flow, affirms the effective regulation methods, and continues to use them in the next cycle regulation; the ineffective regulation methods are analyzed to find out the root causes, and the improvement scheme is discussed again. Analyze the achievements and shortcomings of each cycle regulation, and make targeted strengthening and improvement measures; (3) The inspection stage. The PDCA cycle regulation team does a good job in the inspection of each training to ensure that every nurse completes the relevant training within a specified period of time, and examines the nurses regularly, and the assessment results are linked to rewards and punishments. Evaluate the quality regulation of each workflow in accordance with the regulatory objectives of the disinfection and supply center, including recovery and classification regulation, cleaning and disinfection regulation, inspection and packaging regulation, storage and distribution regulation, and equipment maintenance regulation. Collect the feedback of each department, and evaluate the quality regulation effect of each working link according to the opinion. Do a good job in the classification of quality problems. The quality data of unqualified equipment recovery, equipment cleaning and sterilization, and equipment fault treatment are analyzed every month, and the corresponding rectification measures are put forward. Establish a sound reporting system for quality problems, including work defects or errors, damage to valuable equipment, and substandard quality of equipment handling workflow, when serious quality problems occur, they must be reported to the competent department at a higher level, analyze the quality problems, and put forward improvement measures; and (4) The head nurse organizes team members to study the relevant knowledge of PDCA cycle regulation, including regulation concepts, regulation steps and implementation measures, and conducts special training for various work processes and links. Develop work manuals according to all work processes of the disinfection and supply center, including staff operation manual, staff training manual, product maintenance manual, and pressure steam sterilizer operation manual, and record the safe operation of the equipment every day. Each group leader randomly checks all the items in 3 to 5 sterilized bags every month.

### 2.3. Methods of Nursing Mark

The group meeting is held once a month to discuss with the group members the problems in the application of nursing signs and the methods of improvement, as well as the design of statistical signs, which are produced and distributed by the request office after filling in the application. The logo design should be eye-catching, reasonable cost, uniform specifications, practical and beautiful, and able to reflect the characteristics of the specialty, in order to improve the quality of nursing management and avoid the occurrence of nursing risks.

#### 2.3.1. Disinfection and Medical Equipment Preparation Signs

Mainly including the concentration and method of preparation of various cleaning enzymes and disinfection solutions in the disinfection supply center, uniformly marked in white letters on a blue background and posted on special soaking buckets and corresponding instruments and equipment.

#### 2.3.2. Safety Warning Signs

The emergency plan is posted on the wall in black letters on a uniform white background so that it can be memorized and, in the event of an emergency, can be implemented immediately in accordance with the regulations to prevent errors and accidents. In addition, next to the autoclave and the cleaning and disinfection machine, the “prevent scalding” care sign is posted in a uniform style with white letters on a black background to strengthen the warning and remind staff to do a good job of self-protection.

#### 2.3.3. Signage for Storage of Sterile Items

Standardize and unify the packaging of sterile items used throughout the hospital and fix rigid signs with white characters on a green background on sterile items storage baskets or shelves to facilitate storage and check distribution to improve work efficiency.

#### 2.3.4. Operational Process Signage

According to the strict division of decontamination area, sterilization area, packaging area, and storage area of sterile articles, and unified with white letters on a green background in each area to post all kinds of routine operation procedures; at the same time, unified with white letters on a green background to post all kinds of instruments and equipment operation specification flow chart on the corresponding instruments and equipment using waterproof self-adhesive paper, so as to facilitate standardized operation.

### 2.4. Observation Index

The main results are as follows: (1) the job satisfaction questionnaire made by the disinfection and supply center of our hospital was adopted to evaluate the nurses' satisfaction with the regulation work. The contents of the scale included regulation quality, safety, operation proficiency, and other dimensions. The evaluation grade is assigned into very satisfactory, relatively satisfactory, acceptable, and unsatisfactory. Satisfaction = very satisfactory rate + relatively satisfactory rate; (2) to compare the differences in nursing staff's safety awareness, comprehensive operation skills, and cleaning effect before and after the implementation of nursing safety concept education. The safety awareness score form is self-made by our hospital, and is evaluated from the aspects of safety identification ability, risk prevention consciousness, and service consciousness. The full score is 10, and the higher the score, the better the safety awareness. The evaluation of comprehensive operation skills includes theoretical assessment and operation assessment, with a full score of 100. The better the score, the better the comprehensive operation skills; (3) the qualified rates of washing, sterilization, packaging, and distribution of instruments were compared, and the disinfection quality of instruments was scored and compared. Among them, the qualified rate of washing, sterilization, packaging, and distribution of instruments are evaluated according to the requirements and standards of the instructions for the use of related instruments. The quality of disinfection of instruments and the quality of nursing service were scored by the expert group of the nursing department according to the self-made scale made by our hospital. The results of the pretest indicated that the test-retest reliability coefficient was 0.977 and the internal consistency Cronbach's *α* value was 0.653, which was consistent with the use of this study; (4) the regulation quality before and after the implementation of PDCA cycle regulation was scored by the regulation evaluation scale made by the disinfection and supply center of our hospital, including recovery and classification regulation, cleaning and disinfection regulation, inspection and packaging regulation, and storage and distribution regulation; and (5) to observe the occurrence of adverse events before and after the implementation of PDCA cycle regulation.

### 2.5. Statistical Analysis

SPSS23.0 statistical software was adopted to process the data. The measurement data were presented as ($\bar{x}$ ± *s*). The group design *t*-test was adopted for the comparison and the analysis of variance was adopted for the comparison between multiple groups. Dun-net-*t* test was adopted for comparison with the control group. The counting data were presented in the number of cases and the percentage, *χ*2 test was adopted for comparison between groups, and a bilateral test was employed for all statistical tests.

## 3. Results

### 3.1. Comparison of Quality Evaluation of Nursing Staff

Firstly, we compared the quality evaluation of nursing staff. The quality scores of instrument disassembly, cleaning, disinfection, packaging, and environment in the study group were remarkably higher, and the difference was statistically significant (*P* < 0.05). All the results are indicated in Table 1.

### 3.2. Comparison of Disinfection Qualification of Nurses

We compared the qualified situation of disinfection of nurses. The qualified rates of sterile dry cans, surgical instruments, endotracheal cannula, oxygen humidification bottles, and laryngoscope instruments in the study group were remarkably higher, and the difference was statistically significant (*P* < 0.05). All the results are indicated in Table 2.

### 3.3. Comparison of Quality Regulation Effects

The quality regulation effects were compared. The qualified rate of instrument washing, sterilization, packaging, and distribution in the study group was remarkably enhanced, and the difference was statistically significant (*P* < 0.05). All the results are indicated in Figure 1.

### 3.4. Comparison of Supply Satisfaction

We compared the regulation scores, and the regulation score of recovery and classification regulation, cleaning and disinfection regulation, inspection and packaging regulation, and storage and distribution regulation in the study group were remarkably higher, and the difference was statistically significant (*P* < 0.05). All the results are indicated in Table 3.

### 3.5. Comparison of Scores of Safety Awareness and Comprehensive Operation Skills of Nurses

We compared the scores of safety awareness and comprehensive operation skills. The results of safety identification, risk prevention, service, theory, and operation of nurses in the study group were remarkably higher, and the difference was statistically significant (*P* < 0.05). All the results are indicated in Table 4.

### 3.6. Comparison of Incidence of Adverse Reactions

In the control group, there were 3 complaints, 2 nursing errors, and 1 accident. The incidence of adverse events was 40.00%; there was only one nursing error in the study group, and the incidence of adverse events was 6.67%. The incidence of adverse events in the study group was lower, and the difference was statistically significant (*P* < 0.05). All the results are indicated in Figure 2.

### 3.7. Comparison of Job Satisfaction of Nursing Staff

We compared the job satisfaction of nurses. In the study group, 10 were very satisfied, 2 were relatively satisfied, 1 was satisfied, and no one was dissatisfied, with a satisfaction rate of 92.31%; In the control group, 3 cases were very satisfied, 6 were more satisfied, 3 were satisfied, 1 was not satisfied, and the satisfaction was 53.84%. The satisfaction of the study group was remarkably higher, and the difference was statistically significant (*P* < 0.05). All the results are indicated in Table 5.

## 4. Discussion

With the transformation of the traditional medical model and the implementation of the new medical reform, the requirements of society and medical and nursing service quality are increasing, which makes nursing regulation become particularly vital [16]. Nursing quality regulation is a measure to make the nursing quality reach the best standard under the condition of certain humans. In the meantime, it is also a vital regulation measure to enhance nursing skills. Nursing quality is the overall embodiment of nursing theoretical knowledge, technical level, working attitude, and nursing effect on nursing staff. It is the core content of nursing regulation. And it is closely related to the health and life of patients. The quality of nursing directly affects the overall medical quality. Under the new situation, it has become the primary task of hospital nursing to study how to enhance nursing quality, whose regulation can meet the needs of modern medical development only if it develops in a scientific direction [17].

In some countries, PDCA cycle is widely adopted in various fields of nursing regulation. In the article “using FOCUS-PDCA to solve Clinical Nursing problems,” RedickEL pointed out that FOCUS-PDCA is a systematic, logical, and accurate regulation method for solving complex or multifaceted clinical nursing quality problems [17, 18]. PDCA cycle theory has become one of the effective regulation models for nursing managers. It was presented by Dr. Deming, an American quality regulation expert, in the 1950s. The main content is the abbreviation of Plan, Do, Check, and Action, which is the basic method of TQM. The PDCA cycle can be assigned into four stages: planning stage, implementation stage, inspection stage, and treatment stage [18]. These four stages can often be performed successively. In the actual work, the specific operation is: first set work objectives or ask questions, and then through the analysis of the problems, find out the causes of the problems, and then formulate corresponding measures, implement measures. It is an effective regulation method with continuous improvement and spiral rise [18, 19]. The final aim of the regulation is to optimize various works. PDCA cycle mode accords with the objective law of “practice-cognition-re-practice-re-cognition” and embodies scientific epistemology. So PDCA cycle is taken as a practical regulation philosophy [19]. This scientific regulation procedure was first applied to enterprise regulation and achieved good results. Because of its rigorous operating procedures and diverse regulation levels, PDCA cycle is suitable for different kinds of regulation. It is taken as an effective method to strengthen internal regulation in various industries, and it is also appropriate for all aspects of regulation [19, 20].

Since the 1990s, with the cooperation of nursing experience, nursing regulation in China has become one of the vital contents of medical and health reform. Nowadays, China has made some progress in nursing theoretical and practical research. More managers apply modern regulation theory to nursing quality regulation and put it into practice [21]. In the article “intravenous injection of antibiotics with FOCUS-PDCA,” Demirel et al. pointed out that by constantly modifying, updating, and perfecting the policies of medical institutions and changing nursing processes and measures, the risk of intravenous injection of antibiotics in home nursing was remarkably reduced [22]; Zhou et al. adopted PDCA circulation in the nursing care of patients with severe craniocerebral injury, and Demirel et al. used PDCA circulation in the formulation of the patient care plan to make it more consistent with the patient's condition [23]; The PDCA cycle is also applied to all-round education of nurses and home care of patients. In the nursing field in China, with the unremitting penetration and influence of the concept of PDCA cycle, many nursing researchers in China have applied this theory to the regulation of nursing quality, but there is still a lack of empirical research in disinfection centers [24].

In recent years, with the enhancement of society and the continuous improvement of people's living standards, people's requirements for the quality of the disinfection of food and articles are also increasing, and the work of disinfection and supply center has made great progress. However, there are often irregularities in the preparation of disinfectant solutions, inconsistencies in the assembly of instruments, and a lack of staff knowledge. Some studies have shown that the use of nursing signs serves as a warning to health care staff, thus contributing to a greater awareness of risk among nursing staff. Some research scholars have concluded that the addition of nursing signs to the ward resulted in a significant reduction in the incidence of nursing errors and a significant increase in the accuracy of medication dispensed. Therefore, the application of nursing signs in safe nursing management care is of great significance. Nursing signage management interventions facilitate the professional upgrading of staff expertise. In addition, the sterile supply nursing logo should be centralized after can promote the standardization and proletarianization of safety management work, enhance the staff's awareness of active checking, and improve work efficiency. The application of nursing signs in the nursing safety management of sterilization supply centers helps to standardize the operational processes of staff, improve self-learning awareness enhancement and improve work quality and efficiency.

The hospital sterilization and supply center are responsible for sterilization and sterilization work and also needs to place and equip all kinds of items in order to facilitate the use of dressings, medical supplies, and sterile equipment in each department [25]. However, there are still some defects in the work of the hospital disinfection supply center, such as lack of professional knowledge of nurses, lack of safety awareness, and unskilled operation skills, which will affect the quality of disinfection regulation of the supply center [26]. As a centralized place for hospital disinfection and sterilization and the turnover of aseptic articles, the work efficiency of the disinfection and supply center is directly related to the efficient operation of various departments of medical institutions, and its regulation quality of instruments is an important embodiment of medical and nursing quality [27]. It is directly related to the medical level of the hospital, poor disinfection regulation quality can lead to a hospital infection, and medical disputes, and have a serious adverse impact on the social influence of the hospital [28]. Under the new situation of the sustained and rapid development of the disinfection supply center, it is extremely important to strengthen the nursing regulation of the disinfection supply center, and it is also an issue widely concerned by hospital administrators at present [29]. In their research, Zeng and Wang proposed to carry out a full-process 3C high-quality nursing service model in the disinfection and supply center, which can remarkably enhance the efficacy of instrument disinfection and reduce the incidence of infection; however, the focus of its research is still to promote the working skills of nurses in the disinfection and supply center, and does not elaborate on the importance of nursing logo [30]. Zhu proposed that attention should be paid to the role of nursing signs in the nursing safety regulation of disinfection and supply centers, especially to remarkably reduce the incidence of nosocomial infection [31]. Through the summary of clinical practice for many years, this study also found that a reasonable and eye-catching nursing logo is not only a simple marking and identification but also enables nurses to identify related items quickly and efficiently. To ensure that nurses can accurately and accurately judge whether the items are qualified or not, so as to ensure that the work of the disinfection supply center can be carried out smoothly.

The work of the disinfection and supply center is not only a high-quality completion of disinfection and sterilization, but also undertakes a lot of disinfection work in the hospital, so it is necessary to enhance the work efficiency while improving the quality. Although the routine nursing work is orderly, the steps are cumbersome and lack of necessary identification, resulting in nurses' urgent need for related disinfection equipment cannot being identified. At present, the regulation effect of the hospital disinfection and supply center is not very satisfactory. In order to solve this problem, the disinfection and supply center of our hospital began to apply the PDCA cycle regulation combined nursing label in 2020. Based on the evaluation and analysis of the current regulatory situation of the disinfection and supply center, the quality control strategy was formulated to regularly carry out professional knowledge, skills, and sudden infection to the staff of the disinfection and supply center. Prevention and handling skills training, improve staff's working ability and self-protection awareness, and assess the training results, increase employees' sense of responsibility and motivation, make them work in strict accordance with operating procedures and norms, ensure work quality and efficiency. PDCA cycle implements the inspection mechanism of random inspection by head nurses and regular inspection by the quality control team, actively deals with the results of rewards and punishments, actively adopts the opinions of various departments, and revises the work of the disinfection and supply center. According to the PDCA cycle method to find and solve problems and constantly summarize the work experience to enhance the work quality of the disinfection supply center.

It was found that the quality scores of instrument disassembly, cleaning, disinfection, packaging, and environment in the study group were remarkably higher, and the difference was statistically significant (*P* < 0.05). The qualified rate of disinfection of sterile dry cans, surgical instruments, endotracheal cannula, oxygen humidification bottles, and laryngoscope instruments in the study group was remarkably higher, and the difference was statistically significant (*P* < 0.05). The qualified rates of washing, sterilization, packaging, and distribution of instruments in the study group were remarkably enhanced, and the difference was statistically significant (*P* < 0.05). The score of recovery and classification regulation, cleaning and disinfection regulation, inspection and packaging regulation, storage and distribution regulation in the study group were remarkably higher, and the difference was statistically significant (*P* < 0.05). The nurses' safety identification ability, risk prevention consciousness, service consciousness, theoretical achievement and operation performance in the study group were remarkably higher, and the difference was statistically significant (*P* < 0.05). Based on the analysis of this, PDCA cycle regulation is an innovative regulation mode on the basis of conventional regulation, which promotes the development of nursing quality regulation in the disinfection supply center to a scientific and standardized direction. The PDCA cycle regulation method includes four stages: planning, implementation, inspection, and summarization. Firstly, it analyzes the problems existing in the quality regulation process of the disinfection supply center, defines the regulation objectives, and draws up regulation plans and measures, which realize the procedure and standardization of the regulation of the disinfection supply center, so as to urge every nurse in the disinfection supply center to carry out in accordance with the relevant quality regulation standards. After defining the plan and goal, the nurses completed each work in a planned and purposeful way according to the relevant requirements, which not only enhanced the nurses' regulations consciousness but also promoted their work enthusiasm and initiative. PDCA cycle can find the problems in the supervision process in time and take targeted improvement measures to ensure the continuous improvement of nursing quality in the disinfection supply center. The results indicated that compared to before implementation, the incidence of adverse events after implementation was lower, and the job satisfaction of nurses after implementation was higher, and the difference was statistically significant (*P* < 0.05). This indicates that the implementation of PDCA circulation regulation method in the regulation of disinfection and supply center can effectively prevent and control the occurrence of adverse events such as complaints, nursing errors and accidents, and make all nurses participate in the regulation, which greatly enhances the job satisfaction of nurses. We followed the methods of Ma et al. The same idea can be found in the study put forward by Ma et al. [32]. They have applied new methods in the study, and the conclusions drawn can also give some support to this study.

In summary, the implementation of the PDCA cycle supervision method in the supervision of the sterile supply center in conjunction with the nursing logo is conducive to improving the quality of supervision and sterilization of all work aspects of the sterile supply center, reducing the occurrence of adverse nursing events and promoting the job satisfaction of nurses. In addition, it is conducive to standardizing the operational processes of staff, improving self-learning awareness enhancement, and improving work quality and efficiency. This study still has some shortcomings. Firstly, the quality of this study is limited due to the small sample size we included in the study. Secondly, this research is a single-center study and our findings are subject to some degree of bias. Therefore, our results may differ from those of large-scale multicenter studies from other academic institutes. This research is still clinically significant and further in-depth investigations will be carried out in the future.

## Figures and Tables

**Figure 1:** comparison of quality regulation effects between the two groups.

**Figure 2:** Comparison of the incidence of adverse reactions between the two groups.

**Table 1:** Comparison of quality evaluation of nursing staff [$\bar{x}$ ± *s*].

Grouping	*N*	Instrument disassembly and assembly	Cleaning	Disinfection	Packing	Environment
Control group	13	95.23 ± 2.07	92.41 ± 1.65	94.26 ± 1.93	96.23 ± 2.53	96.84 ± 1.56
Research group	13	80.38 ± 2.16	81.07 ± 2.08	80.57 ± 2.35	82.66 ± 2.01	82.56 ± 2.34
*t* value		19.224	16.542	17.436	16.265	19.666
*P* value		<0.05	<0.05	<0.05	<0.05	<0.05

**Table 2:** Comparison of disinfection qualification of nurses (*n*(%)).

Grouping	*N*	Project	Aseptic dry tank	Surgical instruments	Endotracheal cannula	Oxygen humidification bottle	Laryngoscope
Control group	13	Number of spot checks	200	230	100	100	104
		Qualified times	192 (96.00)	226 (98.26)	100 (100.00)	100 (100.00)	96 (92.31)

Research group	13	Number of spot checks	220	200	76	80	90
		Qualified times	170 (77.27)	150 (75.00)	54 (71.05)	62 (77.50)	66 (73.33)

*χ* ^2^			30.868	8.879	27.273	25.000	12.611
*P*			<0.05	<0.05	<0.05	<0.05	<0.05

**Table 3:** Comparison of regulation scores [$\bar{x}$ ± *s*].

Grouping	*N*	Satisfaction with goods distribution	Satisfaction with goods recovery	Communication satisfaction of department	Service satisfaction
Control group	13	95.18 ± 2.51	97.19 ± 2.14	96.46 ± 2.77	97.23 ± 2.16
Research group	13	86.44 ± 2.25	87.14 ± 2.15	85.89 ± 2.31	84.58 ± 2.21
*t* value		10.042	12.831	11.350	15.854
*P* value		<0.05	<0.05	<0.05	<0.05

**Table 4:** Comparison of scores of safety awareness and comprehensive operation skills of nurses [$\bar{x}$ ± *s*, Points].

Grouping	*N*	Security identification capability	Risk prevention consciousness	Service consciousness	Theoretical achievement	Operation result
Control group	13	9.07 ± 1.31	9.26 ± 1.55	9.56 ± 1.12	97.81 ± 5.73	97.21 ± 5.32
Research group	13	6.94 ± 1.58	7.28 ± 0.94	7.38 ± 1.44	92.64 ± 4.63	91.63 ± 4.85
*t* value		4.019	4.230	4.840	2.718	3.002
*P* value		<0.05	<0.05	<0.05	<0.05	<0.05

**Table 5:** Comparison of job satisfaction of nurses (*n*(%)).

Grouping	*N*	Very satisfied	Be satisfied with	Still can	Not satisfied	Satisfaction
Control group	13	10 (76.92)	2 (15.38)	1 (7.69)	0 (0.00)	12 (92.31%)
Research group	13	3 (23.07)	6 (46.15)	3 (23.07)	1 (7.69)	7 (53.84%)
*χ* ^2^						4.887
*P*						<0.05

## Data Availability

The datasets used and analyzed during the current study are available from the corresponding author upon reasonable request.
